The article "Ascertaining the Prevalence of Group B Streptococcal Infection in Patients with Preterm Premature Rupture of Membranes: A Cross-Sectional Analysis from Pakistan" was retracted in 2021. Reason: plagiarism.

# Ascertaining the Prevalence of Group B Streptococcal Infection in Patients with Preterm Premature Rupture of Membranes: A Cross-Sectional Analysis from Pakistan

**DOI:** 10.7759/cureus.13395

**Published:** 2021-02-17

**Authors:** Saiqa Yaseen, Shumaila Asghar, Irum Shahzadi, Abdul Qayyum

**Affiliations:** 1 Obstetrics and Gynaecology, Lady Willingdon Hospital, Lahore, PAK; 2 Obstetrics and Gynaecology, Sir Ganga Ram Hospital, Lahore, PAK; 3 Pediatric Surgery, Fatima Memorial Hospital, Lahore, PAK

**Keywords:** preterm premature rupture of membrane (pprom), group b streptococcus (gbs)

## Abstract

Introduction

Literature has shown varying results regarding the presence of group B Streptococcal (GBS) infection in pregnant females with preterm premature rupture of membranes (PPROM). The infection can be detrimental to maternal and neonatal well-being. There is a lack of studies that showed the extent of this problem in the local population of Pakistan. Our study aims to determine the frequency of GBS infection in females with PPROM.

Methods

This cross-sectional study was conducted at the Department of Obstetrics & Gynecology, Lahore General Hospital, Pakistan for six months. Informed consent was obtained from each patient. Demographic data were also recorded. Then the amniotic fluid sample was taken during a vaginal examination and was sent to the laboratory of the hospital for assessment of the presence or absence of GBS. Reports were assessed for GBS infection. Baseline demographics including age, body mass index (BMI), parity, and gestational age were presented as mean and standard deviation. Categorical data like parity and GBS infection were presented as frequency and percentage.

Results

The mean age of women was 30.04 ± 6.75 years. The mean gestational age of patients was 34.51 ± 1.75 weeks. Among 150 women, GBS infection was diagnosed in 24 (16%) patients. The occurrence of GBS infection was significantly associated with the age and parity status of women (p < 0.05). However, it was not significantly associated with gestational age and BMI of women (p > 0.05).

Conclusion

Our study showed a low prevalence of GBS infection in females presenting with PPROM. Nonetheless, the presence of infection can lead to detrimental outcomes including neonatal and maternal sepsis. The rate and risk factors of maternal and neonatal GBS colonization may vary in different communities. These rates, as well as the incidence of neonatal disease, need to be thoroughly evaluated to develop appropriate strategies for prevention.

## Introduction

Preterm premature rupture of membranes (PPROM) refers to the rupture of the membranes before the onset of labor in women with less than 37 weeks of gestation age [1]. The dreaded complications of PPROM are responsible for approximately 30% of preterm births [2,3]. In many circumstances, immediate delivery of the baby becomes a necessity to prevent neonatal sepsis in PPROM [1]. However, it is related to an increased risk for respiratory distress syndrome and cesarean delivery rates which may compromise maternal and neonatal well-being [4,5]. The risk factors of PPROM include poor maternal nutrition, smoking, incompetent cervix, and infections [6].

The article "Ascertaining the Prevalence of Group B Streptococcal Infection in Patients with Preterm Premature Rupture of Membranes: A Cross-Sectional Analysis from Pakistan" was retracted in 2021. Reason: plagiarism.

Group B Streptococcus (GBS) colonization among pregnant women is significantly correlated with gestational age, PPROM, and preterm labor [7]. In pregnancy, GBS colonization may cause a varying spectrum of diseases ranging from asymptomatic bacteriuria, urinary tract infections (UTI), to more severe puerperal infections with amnionitis, endometritis, and sepsis [8]. Maternal colonization with GBS in the genitourinary or gastrointestinal tracts is the primary risk factor for disease [9]. These factors make GBS colonization a cause of significant concern especially in women presenting with PPROM.

There is conflicting literature regarding the prevalence of GBS colonization in patients with PPROM. A multitude of various studies has reported the prevalence to be hovering around 11%-25% [6,7,10]. Moreover, there is a lack of data regarding the actual prevalence of GBS colonization in females with PPROM in developing countries which makes the topic an area of active medical research especially in a developing country like Pakistan.

International studies confirmed the presence of GBS colonization in pregnant females presenting with complications of PPROM [7-10]. We planned to conduct this study because this infection can transmit to the neonate and cause hazardous consequences such as neonatal sepsis. The current study aims to assess the prevalence of GBS colonization in females with PPROM. Additionally, we also aim to assess significant demographic associations with GBS infection. Lastly, we also aim to provide recommendations to prevent the infection and its deleterious complications. Our study may aid to improve the practices and guidelines to plan screening, preventive, and management protocols in such females to have better obstetrical outcomes without the risk of the life of the mother as well as a neonate.

## Materials and methods

This cross-sectional study was conducted at the Department of Obstetrics & Gynecology, Lahore General Hospital, Lahore. A total of 244 females presenting with PPROM, gestational age less than 37 weeks (on last menstrual period), and duration of rupture ≤ 13 hours were included in the study via consecutive sampling technique. Females with a chronic systemic disease like pregnancy-induced hypertension (BP ≥ 140/90 mmHg), diabetes (BSR > 186 mg/dl), cardiac abnormalities (abnormal electrocardiography and medical record), recent UTI, and with a history of GBS infection in a previous pregnancy were excluded.

The article "Ascertaining the Prevalence of Group B Streptococcal Infection in Patients with Preterm Premature Rupture of Membranes: A Cross-Sectional Analysis from Pakistan" was retracted in 2021. Reason: plagiarism.

After the application of the exclusion criteria, a total of 150 cases were enrolled in the study. Informed consent was obtained from each patient. Demographic data (including name, age, gestational age, and parity) was also be recorded. Then the amniotic fluid sample was taken during a vaginal examination and was sent to the laboratory for the culture of GBS. Reports were labeled as GBS positive if more than 10 bacteria were detected on high power field (HPF). All the information was collected on a specially designed proforma. All females received standard treatment protocol for PPROM.

All the collected data was entered and analyzed through Statistical Package for Social Sciences, version 20 (SPSS Inc, Chicago, Illinois). Quantitative data like age, body mass index (BMI), parity, and gestational age were presented as mean and standard deviation. Qualitative data like parity and GBS infection was presented as frequency and percentage. Data was stratified for age, gestational age, parity, BMI status to deal with effect modifiers. A chi-square test was applied to assess a significant association between the study variables. A p-value of less than 0.05 was considered statistically significant.

## Results

The present study involving 150 cases, the mean age of patients was 30.04 ± 6.75 years with a range of 18 to 40 years. Mean gestational age was 34.51±1.75 weeks, ranging from 32 and 37 weeks respectively. The baseline characteristics of the study participants are shown in Table 1.

**Table 1:** Baseline characteristics of the study participants

Variable		Mean ± Standard deviation/Range
Age (years)	Mean	30.04 ± 6.75
	Range	18-40
Gestational Age (weeks)	Mean	34.51±1.75
	Range	32-37
Body Mass Index (kg/m^2^)	Mean	25.14±2.77
	Range	20-30.7

Among 150 women, 27 (18%) were nulliparous and 46 (30.7%) were primary parous and the remaining 77 (51.33%) were multiparous. The parity of the study participants is elucidated in Table 2.

**Table 2:** Parity status of the study participants

Parity	Frequency	Percent
0	27	18.0%
1	46	30.7%
2	38	25.3%
3	26	17.3%
4	13	8.7%
Total	150	100.0%

Out of 150 females, GBS infection was diagnosed in 24 (16%) patients while 126 (84%) had no GBS. The frequency of GBS infection was highest in between 34-40 years of age followed by women who were 26-33 years of age and the lowest frequency of GBS infection was seen in women who were in the age group 18-25 years of age. The frequency of GBS infection was significantly higher in women in the higher age group (p = 0.033). This is shown in Table 3.

The article "Ascertaining the Prevalence of Group B Streptococcal Infection in Patients with Preterm Premature Rupture of Membranes: A Cross-Sectional Analysis from Pakistan" was retracted in 2021. Reason: plagiarism.

**Table 3:** Cross-tabulation of group B Streptococcus (GBS) infection with age groups

Age groups	GBS		Total
	Yes	No	
18-25	3 (12.5%)	43 (34.1%)	46
26-33	8 (33.3%)	46 (36.5%)	54
34-40	13 (54.2%)	37 (29.4%)	50
Total	24	126	150

Gestational age of women was not significantly associated with the frequency of GBS infection (p = 0.412). This is delineated in Table 4.

**Table 4:** Cross-tabulation of group B Streptococcus (GBS) infection with gestational age

Gestational Age	GBS		Total
	Yes	No	
32-34	14 (58.3%)	62 (49.2%)	76
35-37	10 (41.7%)	64 (50.8%)	74
Total	24	126	150

Parity was significantly associated with GBS infection. The highest frequency of GBS infection was seen in women with parity 1-2 (p = 0.023). This is shown in Table 5.

**Table 5:** Cross-tabulation of group B Streptococcus (GBS) infection with parity

Parity	GBS		Total
	Yes	No	
0	1 (4.2%)	26 (20.6%)	27
1-2	12 (50%)	72 (57.1%)	84
3-4	11 (45.8%)	28 (22.2%)	39
Total	24	126	150

BMI of women did not show any statistically significant association with GBS infection (p = 0.221). This is elucidated in Table 6.

**Table 6:** Cross-tabulation of group B Streptococcus (GBS) infection with body mass index (BMI)

BMI	GBS		Total
	Yes	No	
Normal	3 (12.5%)	35 (27.8%)	38
Over Weight	21 (87.5%)	89 (70.6%)	110
Obese	0 (0%)	2 (1.6%)	2
Total	24	126	150

## Discussion

GBS has been attributed as the most common bacteria that leads to neonatal sepsis [11,12]. The vertical transmission of GBS most commonly occurs via the maternal genitourinary or gastrointestinal tract colonization, which generally occurs after rupture of membranes or onset of labor [11]. The time between rupture of membranes and delivery is a known risk factor for increased risk of neonatal GBS sepsis and women who undergo expectant management strategy have a longer time to delivery compared with women in whom labor is induced immediately [12].

In our study, out of 150 patients, GBS infection was diagnosed in 24 (16%) patients. A study reported that nearly 25% of the females presenting with PPROM had GBS colonization [6]. Another study delineated the prevalence to be at a dismal 19.5% [7]. A recent study also showed that the frequency of GBS among females presenting with PPROM was 14% only [1]. While an earlier study reported its prevalence to be as low as 10.8% [10]. The dismal outcomes of GBS colonization in PPROM can only be prevented if the variable prevalence among different communities is evaluated. The GBS colonization may lead to sepsis in the mother and the neonate leading to an increased maternal and neonatal mortality rate especially in a developing country [6-8]. Thus there is a need for appropriate timely GBS screening of patients with PPROM. 

The article "Ascertaining the Prevalence of Group B Streptococcal Infection in Patients with Preterm Premature Rupture of Membranes: A Cross-Sectional Analysis from Pakistan" was retracted in 2021. Reason: plagiarism.

Recently, the association of maternal GBS colonization with preterm labor has become a subject of controversy. In 1996, the Centers for Disease Control and Prevention (CDC) attributed preterm delivery as a risk factor for GBS sepsis and recommended the use of prophylactic antibiotics in preterm labor [9]. A study demonstrated that women with heavy GBS colonization at the time of delivery are more likely to deliver their baby prematurely [13]. Another study also showed an association of preterm birth with GBS colonization [14]. On the contrary, other investigators reported no association between preterm labor and cervicovaginal GBS colonization [15,16]. The prevalence of maternal colonization varies in countries owing to socioeconomic and ethnic differences [14,17].

A study from Iran reported that colonization was detected in 9.2% of all mothers [18]. Although GBS colonization was found more frequently in preterm than term patients (12 v/s 7 cases), the difference was not statistically significant [18]. Furthermore, the literature augments and supports the increased risk of preterm labor in women with increasing age [17,18]. In our study, it was also found that women in the higher age group showed a high frequency of GBS infection as compared to lower groups. This can be due to more frequent conditions for contamination these women experience over time. Moreover, the researchers from Iran have also delineated no significant association of GBS infection with gravidity and parity [18] which is consistent with the results of our study. On the contrary, another study showed that multiparity was associated with a lower colonization rate [17]. The differences in colonization rates depend on the particular population and especially on the laboratory methods used to identify GBS [19]. The additional tests performed in our study may account for the lower frequency of colonization in our population in comparison to other developing countries [20].

There is a significantly elevated incidence of early-onset sepsis among mothers and neonates born to mothers with PPROM which requires an assessment of maternal signs of infection and intrapartum fetal monitoring [19,21]. The use of intrapartum fetal monitoring is highly limited in a developing country like Pakistan due to the limited financial resources. As a result, the risk of neonatal sepsis significantly increases [21]. There is an utmost need for risk stratification of patients based on their parity, BMI, and age so that prophylactic antibiotics can be administered and the risk of neonatal sepsis is thus reduced. In our study, the patients were given intravenous antibiotics so that vertical transmission can be prevented. 

The article "Ascertaining the Prevalence of Group B Streptococcal Infection in Patients with Preterm Premature Rupture of Membranes: A Cross-Sectional Analysis from Pakistan" was retracted in 2021. Reason: plagiarism.

The use of convenience sampling and having a cross-sectional study design account for a few limitations of our study. Furthermore, a multicentric study would have given an accurate prevalence of GBS colonization among pregnant women. We recommend further case-control studies to be conducted on the topic so that risk factors for GBS infection can be evaluated in patients with PPROM.

## Conclusions

Results of this study showed a low frequency of GBS infection in females presenting with PPROM. The rate and risk factors of maternal and neonatal GBS colonization may vary in different communities. There is an urgent need for curation of specific guidelines for appropriate screening of high-risk patients so that rate of GBS infection can be controlled. These rates, as well as the incidence of neonatal and maternal sepsis, need to be thoroughly evaluated to develop appropriate strategies for prevention. We recommend the conduction of case-control studies to further evaluate the risk factors of GBS infection with PPROM. The use of prophylactic antibiotics may help in preventing adverse outcomes.
